The article "Cognitive Function and Vitamin D Status in the Chinese Hemodialysis Patients" was retracted in 2023. Reasons: signs of a paper mill; compromised peer review; unreliable results or conclusions.

# Cognitive Function and Vitamin D Status in the Chinese Hemodialysis Patients

**DOI:** 10.1155/2022/2175020

**Published:** 2022-09-09

**Authors:** Jing Zhang, Jun Hu, Ru Zhou, Yuzhen Xu

**Affiliations:** ^1^Department of Nephrology, Wannan Medical College Affiliated Yijishan Hospital, Wuhu, Anhui Province 241001, China; ^2^Hemodialysis Center, Wannan Medical College Affiliated Yijishan Hospital, Wuhu, Anhui Province 241001, China; ^3^Department of Rehabilitation, The Second Affiliated Hospital of Shandong First Medical University, Taian, Shandong Province 271000, China

## Abstract

**Objective:**

Vitamin D insufficiency and the cognitive function decline are both common in patients receiving hemodialysis (HD). The present study evaluated the relation between cognitive function and circulating vitamin D levels in HD patients in Wannan Medical College Affiliated Yijishan Hospital, China.

**Methods:**

This study was conducted in 80 patients receiving HD in Wannan Medical College Affiliated Yijishan Hospital. To measure cognitive function, Montreal Cognitive Assessment-Basic (MoCA-B) Chinese Version was used. The 25-hydroxyvitamin D [25(OH)D], which is applied to assess vitamin D status, was tested. One-way ANOVA, Tukey post hoc test, and the correlation and regression analysis were used in this study.

**Results:**

Based on the MoCA-B, cognitive function decline (the scores below 26) was present in 28 HD patients, accounting for 35% (28/80). The mean age of these patients is 50.5 ± 10.9 years old. The mean level of 25(OH)D was 16.1 ± 7.3 ng/ml in 80 HD patients. In univariate analysis, there was a significant relationship between MoCA-B score and serum 25(OH)D level (*p* < 0.05). The level of 25(OH)D was positively correlated with MoCA-B score (*r* = 0.312, *p* = 0.023), and the association was independent of demographic and clinical features.

**Conclusions:**

Vitamin D insufficiency may contribute to cognitive function decline in HD patients. Serum level of 25(OH)D is an independent protective factor of cognitive function in the HD patients.

## 1. Introduction

Chronic kidney disease (CKD) has become a major public health problem worldwide. According to the 2012 national epidemiological survey, the overall prevalence of CKD was 10.8% [1] in China, that is, there are about 130 million patients with CKD in China. CKD are independent risk factors for cognitive dysfunction [2]. Cognitive function decline is common in dialysis patients, with the prevalence of mild to moderate cognitive dysfunction up to 70% in hemodialysis (HD) population [3]. What is more, cognitive dysfunction is an independent predictive factor for all-cause mortality in the patients undergoing HD. Therefore, cognitive function decline will become a more and more serious problem in this population [4].

Vitamin D is a kind of fat-soluble seco-steroid necessity for calcium uptake and bone metabolism [5], which is mainly synthesized in the skin after sun exposure. Vitamin D insufficiency has been reported to be common among patients with CKD [6] because of declined renal function and vitamin D metabolism disorder [7]. Vitamin D insufficiency has also been related to many statuses, such as obesity, cardiovascular, and neurodegenerative diseases [8, 9]. Some literatures have demonstrated that vitamin D is closely related to cognitive function decline [10, 11]. Therefore, vitamin D insufficiency is considered as a potentially reversible hazard factor of declined cognitive function. However, little is known about the relationship between the level of vitamin D and the cognitive function in HD patients of China.

25-Hydroxyvitamin D [25(OH)D] (with a half-life of 2-3 weeks [12]) is a metabolite of vitamin D and is also considered as the main circulating form of vitamin D. It is widely applied to assess vitamin D status. Thus, in this study, our purpose is to assess the association between 25(OH)D level and cognitive function in HD patients at a single hemodialysis center.

## 2. Patients and Methods

### 2.1. Study Population

All the HD participants (from Wannan Medical College Affiliated Yijishan Hospital) were patients aged 30–82 years who were receiving HD more than 6 months. The study was approved by the Ethics Committee of Yijishan Hospital Affiliated to Wannan Medical College. The written approval consents from participants and/or their guardians were obtained prior to enrollment in the study. Exclusion criteria were: age < 18years or >90years; HD vintage < 6months; suffered from dementia, cerebrovascular disease, infection, or other serious illnesses such as malignancy during the 6 months before the study; unable or unwilling to answer the questionnaire. None of the patients had taken vitamin D during the study.

### 2.2. Hemodialysis

All the patients were receiving conventional HD (thrice weekly, 4 h each time) through autologous arteriovenous fistula and used “Gambro” HD machine, “Gambro” Polyflux L capillary dialyzers, and bicarbonate dialysate. The blood flow ranged from 220 to 260 ml/min with a dialysate flow of 500 ml/min. All the patients were injected intravenously with low molecular heparin before HD for anticoagulation, according to body weight (60-80 IU/kg). All of them were treated with recombinant human erythropoietin (rhEPO) according to their anemia status and L-Carnitine after each session of HD.

### 2.3. Laboratory Measurements

The clinical, laboratory tests in HD patients were performed at the beginning of the study. Blood for assessment of biochemical characteristics were collected from the HD patients, after fasting for more than 8 hours. The isolated serum samples were measured for the biochemical parameters, such as albumin, blood glucose, renal function (including blood urea nitrogen and serum creatinine), lipids profiles (including total cholesterol, triglycerides, high-density lipoprotein cholesterol, and low-density lipoprotein cholesterol), calcium and phosphorus and intact parathyroid hormone (iPTH), and vitamin D status [25(OH)D].

### 2.4. Cognitive Assessment Examination

The Chinese translation version of MoCA-B test was administered in all participants. The full score of MoCA-B test is 30, and a score below 26 is indicative of cognitive function decline. The testing personnels have been trained by the neurologist.

### 2.5. Statistical Analyses

All the data were analyzed by SPSS 22.0 statistical software. The continuous variables were expressed as means (standard deviation), and categorical variables were summarized as numbers and percentages. One-way ANOVA and subsequent Tukey post hoc test were used to analyze the data between the groups. Further, the correlation and regression analyses between demographic, clinical laboratory features, and MoCA-B scores were performed. *p* < 0.05 was regarded as a significant difference.

## 3. Results

The demographic information and clinical laboratory data and MoCA-B scores of patients receiving HD are presented in Table 1. In total, 80 subjects comprising 43 (53.75%) males and 37 (46.25%) females were enrolled to this study, and fortunately, no one dropped out of this research. The average age of the subjects was 52.3 ± 11.1 years old (from 30 to 82 years old). The primary causes contributed to HD are chronic glomerulonephritis, hypertension, and diabetes, accounting for 40%, 10%, and 47.5%, respectively.

In our study, the mean MoCA-B score of all the participants was 26.0 ± 2.0 (ranged between 22 and 30). 28 patients showed cognitive function decline (MoCA − B score < 26), accounting for about 35%. The mean age of those patients with MoCA − B score < 26 is 50.5 ± 10.9 years old. The demographic, laboratory features, and MoCA-B scores of the participants were displayed in Table 2. There was no significant difference in demographic and laboratory features except MoCA-B scores. From Table 2, we can see that the lower the 25(OH)D level, the worse the cognitive function may be.

The Spearman rank correlation test (Table 3) shows MoCA-B score was positively correlated with 25(OH)D (*r* = 0.312, *p* = 0.023). However, MoCA-B score showed no correlation with demographic parameters (such as age, sex, and years of education) and other clinical parameters (such as concentrations of hemoglobin and other biochemical parameters).

Table 4 presented the association of serum 25(OH) D tertiles with MoCA-B scores in the HD patients. After adjusting age, sex, education, smoking, HD duration, and the clinical and laboratory parameters (such as SBP, DBP, Hb, Alb, BUN, Scr, Ca, P, BG, iPTH, TC, TG, HDL-C, and LDL-C), compared with the subjects in tertiles 1 [25(OH)D ≤ 10.77 ng/ml], there was significant protection for cognitive function with the subjects in tertiles 3 [25(OH)D > 19.24 ng/ml] (OR = 2.113; 95% CI 0.971-4.397; *p* = 0.037). The average MoCA-B score (26.0 ± 1.8) of subjects in tertiles 2 [25(OH)D: 10.77–19.24 ng/ml] increased, compared with that in tertiles 1(OR = 2.203; 95% CI 1.732-2.488,p =0.261), but there was no significant statistical difference between two groups (tertiles 1 versus tertiles 2).

## 4. Discussion

In our current study, HD patients had a relative high prevalence of cognitive function decline, and the level of serum 25(OH)D is positively related to the MoCA-B score in the HD population. This relationship was independent of demographic and clinical laboratory features. Our results also demonstrated that the high level of 25 (OH)D in serum was an independent protective factor for predicting good cognitive function in Chinese HD patients.

Cognitive function decline can occur at all stages of CKD, including early stage [13] and end stage [14]. In addition to cardiovascular complications, the neurologic complications are also very prevalent in CKD patients, especially in dialysis patients. One of the neurological complications is cognitive function decline [15], which is remarkably associated with CKD, but not with age and other potential confounders [16]. The cognitive function of HD patients of all ages is worse than individuals of the general population of the same age [3]. In our current study, 35% HD patients appeared cognitive function decline, which is different from our previous study [17] that reported that only 15% HD patients appeared cognitive function decline. The main reason may be lie in the different assessment method and the different primary disease causing end stage renal disease (ESRD). In this study, diabetes was the primary disease in almost half of the HD patients (accounting for 47.5%), whereas this proportion accounted for only 32% in our previous study [17]. In the Miskulin's Cohort Study [18], diabetes is the primary cause in 47% of patients with ESRD, which is similar to this study. Diabetes and ESRD are both independent risk factors for cognitive function decline because advanced glycosylation end-product accumulation may trigger vascular endothelial dysfunction [19] and impaired cerebral blood flow in ESRD, which finally contributed to cognitive function decline. However, there are few studies about the combined impact of diabetes and ESRD on cognitive function. In the future, we will focus on the cognitive function of the patients with diabetic ESRD.

The poor cognitive function is high prevalent in elderly population [13]. The older the age, the greater the decline of cognitive function every year, regardless of sex, race, education, stroke history, or cause of renal failure [20]. However, the result of our study presented differently. The average age of HD patients with cognitive function decline in our study is only 50.5 ± 10.9 years old, which is similar to a seven-year study [21]. In that study, not only elderly but also younger aged dialysis patients (mean age: 51.81 ± 14.05 years old) presented significant cognitive function decline. Therefore, HD patients may have a high risk of cognitive function decline even at younger ages.

The causes of poor cognitive function are not fully understood in the adult population receiving HD, and several factors might be involved in the high prevalence of cognitive function decline and rapid deterioration in HD patients. The uremic toxins has been reported to potentially lead to poor cognitive function, because cognitive function was improved with the restoration of renal function after kidney transplantation [22]. In addition, there are other risk factors between cognitive function decline and ESRD.

Vitamin D is gradually recognized and attached importance because of its effect on cognitive function. Vitamin D levels are decreased in population suffered from mild cognitive impairment [23], and vitamin D insufficiency is a potential risk factor for cognitive function decline in the general population [10]. A part of the reason is that higher circulating levels of 25(OH)D exerts vasculoprotective and neuroprotective properties to improve cognitive function. The mechanism involved in inhibiting proinflammatory factors, antioxidation, immunoregulation, and enhanced nerve conduction [24]. 25(OH)D insufficiency is also associated with endothelial dysfunction [25], which is related to cognitive impairment [26]. An animal experimental study [27] also found that increasing the level of 25(OH)D could prevent the age-related cognitive function decline in aged rats. The reason was that vitamin D was thought to strengthen hippocampal synaptic function in aged rats.

Despite of different subjects, the mean level of serum 25(OH)D is 16.1 ± 7.3 ng/ml in this study, which is similar to the previous report (the mean level of serum 25(OH)D ± SD was 17.26 ± 7.4 ng/ml) [28]. We also found an association between serum low levels of vitamin D [assessed by 25(OH)D] and cognitive function decline in Chinese HD patient, which is also consistent with Kamran's study of HD patients in the United States [28]. In this study, patients with higher 25(OH)D tertile had significantly higher MoCA-B scores. The spearman correlation test shows that the serum 25(OH)D level is positively related to MoCA-B scores (*r* = 0.312; *p* < 0.05). However, not all literatures report such association. A study by Jovanovich et al. [29] of 605 veterans with advanced CKD and chronic dialysis reported that the levels of plasma 25(OH)D could not independently predict TICSm score, a method for measuring cognitive function in advanced CKD and ESRD. This discrepancy may lie in: (1) different investigation methods (face to face questionnaire and telephone survey); (2) different method for measuring cognitive function (MoCA-B and TICSm); (3) different research objects (men and women are almost equally divided and nearly entirely men); (4) racial differences.

Except for the correlation between serum 25(OH)D and MoCA-B scores, previous studies have confirmed the associations between higher SBP and DBP and cognitive impairment in the general population [30]. However, other studies suggested that there was no relationship between changes in SBP or intradialytic change in blood pressure with cognitive function decline [31]. Our study also found there is no relationship between SBP and cognitive function. The main cause may be that the subjects are different. The elevated iPTH levels were associated with impaired cognitive function in the patients suffered from secondary hyperparathyroidism due to calcium deficit rather than renal function impairment [32], whereas nocturnal daily HD improved cognitive function, which may be partly due to reduced iPTH levels [33]. However, we did not find an independent relationship between iPTH levels and cognitive function in HD patients.

In conclusion, serum 25(OH)D affects cognitive function in HD patients. The level of serum 25(OH)D may play independent roles in cognitive function decline. The potential mechanism needs to be further explored.

## 5. Limitations of the Study

There were several limitations in this study. In the first place, the sample of the patient population is relatively small (only 80 patients), which may produce selection bias and made this study underpowered. Thus, it is recommended to expand the sample sizes, and we are convinced that expanding the sample size would more reveal that whether reduced 25(OH)D raises the incidence of cognitive function decline in the HD patients. Second of all, the average age of HD patients is only 52.3 years in this study, which is slightly younger than the present age in many developed populations [34]. Therefore, the results of this study could not represent HD patients in other dialysis centers.

## Figures and Tables

**Table 1:** Demographic information and laboratory data and MoCA-B scores of HD patients (*N* = 80).

Characteristics	Outcomes
Age, yr (range)	52.3 ± 11.1 (30-82)
Males, *N* (%)	43 (53.75)
Females, *N* (%)	37 (46.25)
*Education, yrN(%)*	
0-3	13 (16.25)
3-6	35 (43.75)
6-12	30 (37.5)
>12	2 (2.50)
*Antecedents,N(%)*	
Diabetes	38 (47.5)
Hypertension	8 (10.0)
Glomerulonephritis	32 (40.0)
Others	2 (2.5)
Duration of HD (months)	53.6 ± 26.4
Smokers, *N* (%)	3(3.75)
Predialysis SBP, mmHg	140.2 ± 20.3
Predialysis DBP, mmHg	73.3 ± 9.5
MAP, mmHg	95.6 ± 11.4
MoCA-B score	26.1 ± 2.0 (22-30)
MoCA − B score < 26	
*N* (%)	28 (35)
Age, yr	50.5 ± 10.9
*Clinical laboratory characteristics*	
25(OH)D, ng/ml	16.1 ± 7.3
Hb, g/l	112.6 ± 16.8
Alb, g/l	40 ± 4.4
BUN, mmol/l	24.4 ± 8.4
Scr, *μ*mol/l	877.1 ± 231.3
Ca, mmol/l	2.4 ± 0.2
P, mmol/l	1.7 ± 0.5
BG, mmol/l	5.3 ± 2.0
TC, mmol/l	4.0 ± 1.0
TG, mmol/l	1.7 ± 0.8
HDL-C, mmol/l	1.3 ± 0.3
LDL-C, mmol/l	2.2 ± 0.7
iPTH, pg/ml	317.5 ± 317.4

Continuous variables are expressed as means ± SD, and categorical variables were summarized as numbers (percentages). SBP: systolic blood pressure; DBP: diastolic blood pressure; MAP: mean arterial pressure; 25(OH)D: 25 hydroxyvitamin D; Hb: hemoglobin; Alb: albumin; BUN: blood urea nitrogen; Scr: serum creatinine; Ca: calcium; P: phosphorus; BG: blood glucose; TC: total cholesterol; TG: triglyceride; HDL-C: high-density lipoprotein cholesterol; LDL-C: low-density lipoprotein cholesterol; iPTH: intact parathyroid hormone; mM: mmol/l.

**Table 2:** Demographic, laboratory features, and MoCA-B scores of three groups.

Variable	Tertile 1	Tertile 2	Tertile 3	*p*
25(OH)D(ng/ml)	≤10.77	10.77-19.24	>19.24	—
Age (yr)	53 ± 12.5	49.6 ± 10.6	54.2 ± 9.9	0.206
Male (*n*)	15	12	16	0.624
Female (*n*)	11	15	11	0.569
Education (yr)	6.7 ± 2.4	6.6 ± 2.4	7.0 ± 2.4	0.074
Smokers (*n*)	1	1	1	—
SBP, mmHg	144.2 ± 19.2	145.0 ± 18.0	131.5 ± 21.3	0.097
DBP, mmHg	74.8 ± 11.2	74.9 ± 8.9	70.1 ± 8.2	0.324
Duration of dialysis (months)	48.8 ± 31.5	53.7 ± 24.1	48.4 ± 23.2	0.247
Hb, g/l	113.1 ± 22.2	110.6 ± 15.1	113.9 ± 12.2	0.812
Alb, g/l	39.5 ± 5.4	38.9 ± 4.2	41.7 ± 2.7	0.746
BUN, mmol/l	20.5 ± 5.5	22.1 ± 7.3	20.8 ± 5.6	0.692
Scr, *μ*mol/l	837.0 ± 241.8	853.7 ± 242.1	939.3 ± 203.6	0.186
Ca, mmol/l	2.4 ± 0.2	2.3 ± 0.2	2.4 ± 0.2	0.717
P, mmol/l	1.7 ± 0.4	1.7 ± 0.5	1.7 ± 0.5	0.826
BG, mmol/l	5.3 ± 2.7	5.3 ± 1.9	5.3 ± 1.0	0.844
TC, mmol/l	4.0 ± 1.0	4.0 ± 1.0	3.9 ± 1.0	0.656
TG, mmol/l	1.7 ± 0.7	1.8 ± 1.0	1.6 ± 0.7	0.532
HDL-C, mmol/l	1.3 ± 0.3	1.3 ± 0.3	1.3 ± 0.3	0.781
LDL-C, mmol/l	2.2 ± 0.8	2.2 ± 0.6	2.1 ± 0.7	0.889
iPTH, pg/ml	292.5 ± 253.5	332.1 ± 305.3	326.5 ± 266.9	0.068
MoCA-B score	24.8 ± 1.7	26.0 ± 1.8	27.5 ± 1.7	0.042

25(OH)D: 25-hydroxyvitamin D; SBP: systolic blood pressure; DBP: diastolic blood pressure; MAP: mean arterial pressure; Hb: hemoglobin; Alb: albumin; BUN: blood urea nitrogen; Scr: serum creatinine; Ca: calcium; P: phosphorus; BG: blood glucose; TC: total cholesterol; TG: triglyceride; HDL-C: high-density lipoprotein cholesterol; LDL-C: low-density lipoprotein cholesterol; iPTH: intact parathyroid hormone.

**Table 3:** Correlation analysis between MoCA-B and various parameters.

	*r*	*p*
Age (yr)	0.347	0.231
Male (*n*)	0.376	0.356
Education (yr)	0.221	0.279
Smokers (*n*)	0.768	0.697
SBP, mmHg	0.531	0.133
DBP, mmHg	0.651	0.098
Duration of dialysis(months)	0.257	0.146
Hb, g/l	0.374	0.333
Alb, g/l	0.419	0.103
BUN, mmol/l	0.544	0.265
Scr, *μ*mol/l	0.731	0.247
Ca, mmol/l	0.424	0.421
P, mmol/l	0.537	0.258
BG, mmol/l	0.471	0.394
TC, mmol/l	0.604	0.136
TG, mmol/l	0.495	0.289
HDL-C, mmol/l	0.537	0.686
LDL-C, mmol/l	0.289	0.691
iPTH, pg/ml	0.114	0.218
25(OH)D, ng/ml	0.312	0.023

SBP: systolic blood pressure; DBP: diastolic blood pressure; MAP: mean arterial pressure; 25(OH)D: 25 hydroxyvitamin D; Hb: hemoglobin; Alb: albumin; BUN: blood urea nitrogen; Scr: serum creatinine; Ca: calcium; P: phosphorus; BG: blood glucose; TC: total cholesterol; TG: triglyceride; HDL-C: high-density lipoprotein cholesterol; LDL-C: low-density lipoprotein cholesterol; iPTH: intact parathyroid hormone.

**Table 4:** Association of serum 25(OH) D tertiles with MoCA-B scores.

ORs (95% CI), *p* value			
	Tertile 1	Tertile 2	Tertile 3
*N*	26 1 (reference)	27 2.203 (1.732-2.488), *p* = 0.261	27 2.113 (0.971-4.397), *p* = 0.037

Adjusted for age, sex, education, smoking, duration of HD, SBP, DBP, Hb, Alb, BUN, Scr, Ca, P, BG, iPTH, TC, TG, HDL-C, and LDL-C; SBP: systolic blood pressure; DBP: diastolic blood pressure; Hb: hemoglobin; Alb: albumin; BUN: blood urea nitrogen; Scr: serum creatinine; Ca: calcium; P: phosphorus; BG: blood glucose; iPTH: intact parathyroid hormone; TC: total cholesterol; TG: triglyceride; HDL-C: high-density lipoprotein cholesterol; LDL-C: low-density lipoprotein cholesterol.

## Data Availability

The data used to support the findings of this study are available from the corresponding author upon reasonable request.
